# Clinical Pregnancy and Incidence of Ovarian Hyperstimulation Syndrome in High Ovarian Responders Receiving Different Doses of hCG Supplementation in a GnRH-Agonist Trigger Protocol

**DOI:** 10.1155/2021/2180933

**Published:** 2021-10-25

**Authors:** Xiuzhen Shen, Qinjie Yang, Lanfang Li, Wenhao Lu

**Affiliations:** ^1^Reproductive Center, Taizhou Hospital of Zhejiang Province, Taizhou, China; ^2^Ultrasound Department, Taizhou Hospital of Zhejiang Province, Taizhou, China

## Abstract

**Objective:**

Ovarian hyperstimulation syndrome (OHSS) is a side effect of the exogenous human chorionic gonadotropin (hCG) hormones used to trigger oocyte maturation. High ovarian responders represent a population with a higher risk of OHSS and are characterized by an exaggerated response to gonadotropin administration. In this study, we compared clinical pregnancy and incidence of OHSS in high ovarian responders receiving different doses of hCG supplementation in a GnRH-agonist trigger protocol.

**Methods:**

A total of 205 high ovarian responders who were to undergo in vitro fertilization (IVF)/intracytoplasmic sperm injection (ICSI) cycles were recruited and randomly assigned to receive different doses of hCG supplementation in a GnRH-agonist trigger protocol: GnRH-a (*n* = 42), GnRH-a + 1000 IU hCG (*n* = 49), GnRH-a + 2000 IU hCG (*n* = 54), and GnRH-a + 3000 IU hCG (*n* = 60) groups.

**Results:**

The GnRH-a + 1000 IU hCG, GnRH-a + 2000 IU hCG, and GnRH-a + 3000 IU hCG groups had more oocytes retrieved, embryos, high-quality embryos, and a higher rate of high-quality embryos than the GnRH-a group (*p* < 0.05). The GnRH-a + 1000 IU hCG group demonstrated more oocytes retrieved, embryos, high-quality embryos, and a higher rate of high-quality embryos than the GnRH-a + 2000 IU hCG and GnRH-a + 3000 IU hCG groups (*p* < 0.05). No moderate and severe OHSS cases occurred in the GnRH-a and GnRH-a + 1000 IU hCG groups. The incidence rate of moderate and severe OHSS was remarkably lower in the GnRH-a group and GnRH-a + 1000 IU hCG groups than in the GnRH-a + 2000 IU hCG and GnRH-a + 3000 IU hCG groups (*p* < 0.05). The GnRH-a + 1000 IU hCG, GnRH-a + 2000 IU hCG, and GnRH-a + 3000 IU hCG groups had a higher clinical pregnancy rate than the GnRH-a group, showing no significant difference (*p* > 0.05). The GnRH-a + 1000 IU hCG, GnRH-a + 2000 IU hCG, and GnRH-a + 3000 IU hCG groups had a lower abortion rate than the GnRH-a group (*p* < 0.05).

**Conclusion:**

Based on the data obtained from this prospective study, we recommend 1000 IU hCG supplementation in a GnRH-agonist trigger protocol for high ovarian responders during IVF/ICSI cycles considering a higher rate of high-quality embryos, a lower incidence rate of moderate and severe OHSS, and a lower abortion rate.

## 1. Introduction

Since the birth of the first test tube baby in 1978, assisted reproductive technology (ART), mainly in vitro fertilization embryo transfer (IVF-ET), has become an indispensable part of modern medicine, which contributes to implementing family planning [1]. IVF technology is a complex medical treatment process. While pursuing to improve the clinical pregnancy rate, the professionals are also constantly committed to improving the safety of the treatment and minimizing treatment complications. Since the combination of relatively large and high-quality eggs and sperm is the first step of a successful pregnancy, the selection scheme of controlled ovarian hyperstimulation (COH) is an essential part of treatment [2]. COH aimed at producing more oocytes. Nevertheless, it occasionally leads to ovarian hyperstimulation syndrome (OHSS), which is an iatrogenic syndrome. OHSS is associated with the use of exogenous gonadotropin and characterized by a variety of symptoms, including excessive follicular development of ovarian epithelium, enlarged ovarian volume, increased steroid hormone level in the body, increased vascular permeability, extravasation of protein rich body fluids, electrolyte disorder, and disorder of liver and kidney function and thrombosis, which can be life-threatening in severe cases [3, 4].

In recent years, with the worldwide popularity and the extensive development of IVF-ET, the incidence of OHSS showed an upward trend. It has been estimated, among the females receiving IVF-ET in clinical, the prevalence of mild was approximately 20% to 33%, and the moderate or severe females was nearly 3% to 8% [5]. Females with a high ovarian response, such as ovulation disorders and polycystic ovary syndrome (PCOS), as well as young age and low body mass index, are associated with an increased risk of OHSS [6]. For decades, human chorionic gonadotropin (hCG), which induces luteinization of granulosa cells and triggers final oocyte maturation, has been widely used in COH. However, among females who used hCG for COH, the incidence of moderate OHSS has ranged from 3% to 7%, and the incidence of severe OHSS has reached between 0.1% and 2% [3]. Once OHSS occurs, it will not only increase patients' pain and additional medical expenses but also lead to serious complications and even be life-threatening. With the improvement of clinical and laboratory technology, pretreatment biomarkers have been applied to individualize the dose of exogenous gonadotropin in IVF-ET. Gonadotropin releasing hormone agonists (GnRH-a) has been accepted to prevent the surge of premature luteinizing hormone (LH) [7]. In the last two decades, GnRH-a has been a trigger factor for the final follicle maturation, which significantly reduced the incidence rate of OHSS clinically [8, 9]. However, many studies have reported that GnRH-a trigger protocol is prone to luteal insufficiency [10], resulting in the decrease of clinical pregnancy rate and the increase of early abortion rate [11, 12].

Some researchers suggested that GnRH-a and hCG dual trigger might be associated with improvements in clinical outcomes, involving clinical pregnancy rate and live birth rate per transfer, but the risk of OHSS remains unclear [13, 14]. In the present study, we aimed to evaluate the safety and efficacy of GnRH-a trigger protocol with different doses of hCG in IVF-ET for high ovarian responders. The clinical outcomes, including embryos quality, clinical pregnancy rate, oocytes retrieved numbers, and incidence rate of OHSS, will be analyzed to provide application reference in further clinical research of IVF-ET.

## 2. Methods

### 2.1. Study Participants

High ovarian responders who were to undergo IVF/intracytoplasmic sperm injection (ICSI) cycles in our hospital from January 2016 to January 2021 participated in this prospective longitudinal study. High ovarian responders are defined with serum levels of estradiol >5000 pg/ml on hCG day and/or numbers of retrieved oocytes >15 [15, 16]. The inclusion criteria were as follows: age ranging from 21 to 38 years; basal follicle-stimulating hormone (FSH) level <8 IU/L; basal luteinizing hormone (LH)/FSH ≥2; more than 10 antral follicle count (AFC) by B-ultrasound observation; oligomenorrhea and use of drugs to induce menstruation; hyperandrogenism; diagnosis of polycystic ovary syndrome according to the Rotterdam Criteria in a year; normal uterine appendages; IVF/ICSI. Patients were excluded for the following reasons: history of IVF/ICSI failure due to sperm or fertilization; with endometriosis and adenomyosis; abnormal vaginal bleeding; habitual abortion; previous diagnosis of uterine adhesion; malformation in reproductive system; diameter of ovarian cyst ≥35 mm; hydrosalpinx; presence of autoimmune, endocrine, and metabolic diseases; mental disorder; undergoing blastocyst biopsy for preimplantation genetic testing; ectopic pregnancies; and acute infection of the urogenital system and sexually transmitted diseases. Eligible subjects were randomly assigned to GnRH-a, GnRH-a + 1000 IU hCG, GnRH-a + 2000 IU hCG, and GnRH-a + 3000 IU hCG. The study was approved by the Ethics Committee of the Enze Women's and Children's Hospital Affiliated with Zhejiang Enze Medical Group, and all participants provided written informed consent.

### 2.2. Controlled Ovarian Hyperstimulation (COH) Protocols

On the third day of the menstrual cycle, 112.5–150 IU/day of Gn was first given, followed by administration of an antagonist (cetrorelix, Merck, Switzerland or ganirelix, MRK, Netherlands) at the dose of 0.125 mg–0.25 mg/day when the follicular diameter reached 14 mm in 1 ovarian follicle or 13 mm in 2 ovarian follicles; the LH level reached ≥10 m IU/ml, or estradiol ≥1000 pg/ml. Once the follicular diameter reached 18 mm in ≥1 ovarian follicle, 17 mm in ≥2 ovarian follicles, or 16 mm in ≥3 ovarian follicles, there was a subcutaneous injection of 0.2 mg GnRH-a alone or in combination with intramuscular injection of 1000 IU hCG, 2000 IU hCG, or 3000 IU hCG.

### 2.3. Oocyte Retrieval and IVF/ICSI-Frozen Embryo Transfer (FET)

Thirty-six hours later, oocyte retrieval was performed by transvaginal ultrasound-guided aspiration. After preparing the husband's sperms or frozen sperms, IVF/ICSI was performed according to the number and quality of sperms, with retrieved oocytes and mature oocytes calculated. Normal fertilization was defined as the presence of 2 pronuclear in the oocyte cytoplasm. The high-quality embryos included grade I and grade II day 3 embryos according to grading system [17]—grade I: the blastomeres had even sizes, regular shapes, and intact zona pellucida, with cell debris rate less than 10%; grade II: the blastomeres had slightly irregular morphology, and the cytoplasm might have granulation, with cell debris rate between 10 and 20%; grade III: the blastomeres were uneven in size and irregular in shape, and the cytoplasm had obvious granulation, with cell debris rate between 20 and 50%; and grade IV: the blastomeres were severely uneven in size and severely irregular in shape, and the cytoplasm had a lot of granulation, with cell debris rate more than 50%. One day after oocyte retrieval, normal embryos were counted. On the third day following oocyte retrieval, high-quality embryos were counted, and the occurrence and severity of OHSS were evaluated according to leukocyte counts, hematocrit, hepatic enzymes, ovarian size measurement by B-ultrasound, ascites, pleural effusion, and uncomfortable symptoms of the patients. The severity of OHSS was graded as mild, moderate, and severe [18]. FET was performed concerning poor endometrial receptivity or incidence of moderate and severe OHSS. In this study, all participants underwent FET. According to participants with or without spontaneous ovulation, endometrial preparation protocols including hormone replacement cycles, ovulation induction cycles, or downregulation hormone replacement cycles were performed for FET. When the thickness of the endometrium reached more than 8 mm, progesterone 60 mg/d was injected intramuscularly to transform the endometrium, and the FET was performed 3 days later.

### 2.4. Outcome Variables

The primary outcome measures were the number of retrieved oocytes, the rate of fertilization, the number of high-quality embryos, the rate of clinical pregnancy, the abortion rate, and the incidence rate and severity of OHSS. Clinical pregnancy was defined as the ultrasonographic visualization of one or more gestational sacs or a fetal heartbeat 4–6 weeks after ET.

### 2.5. Data Analyses

Continuous variables are expressed as mean ± standard deviation and compared by one-way analysis of variance. Categorical variables are expressed as proportions and analyzed using the chi-square test or Fisher's exact probability method. SPSS 22.0 software was employed to perform data management and analysis. *p* < 0.05 is considered statistically significant.

## 3. Results

### 3.1. Baseline Characteristics of Study Participants

Figure 1 shows participant flow and study design. A total of 205 high ovarian responders meeting the inclusion and exclusion criteria were recruited and randomly assigned to GnRH-a (*n* = 42), GnRH-a + 1000 IU hCG (*n* = 49), GnRH-a + 2000 IU hCG (*n* = 54), and GnRH-a + 3000 IU hCG (*n* = 60) groups. In the GnRH-a group, the women had a mean age of (30.57 ± 4.47) years and a mean infertility duration of (4.29 ± 2.06) years, and their infertility causes were pelvic factors (*n* = 16), ovulation dysfunction (*n* = 12), tubal factors (*n* = 9), and other factors (*n* = 5). The GnRH-a + 1000 IU hCG group had a mean age of (30.65 ± 4.39) years and a mean infertility duration of (4.41 ± 2.33) years, including 19 cases due to pelvic factors, 14 cases due to ovulation dysfunction, 10 cases due to tubal factors, and 6 cases due to other factors. The GnRH-a + 2000 IU hCG group with a mean age of (29.30 ± 4.26) years and a mean infertility duration of (3.89 ± 2.59) years consisted of 22 cases of pelvic factors, 15 cases of ovulation dysfunction, 11 cases of tubal factors, and 6 cases of other factors. With regard to the GnRH-a + 3000 IU hCG group, the women had a mean age of (30.32 ± 4.07) years and a mean infertility duration of (3.72 ± 2.05) years, and their infertility causes were pelvic factors (*n* = 23), ovulation dysfunction (*n* = 18), tubal factors (*n* = 12), and other factors (*n* = 7). The information about basal FSH, basal LH, basal estradiol, AFC, duration of Gn stimulation, and total dosage of Gn of all participants are listed in Table 1. No significant difference was noted in the mean age, infertility duration, infertility causes, basal FSH, basal LH, basal E2, AFC, duration of Gn stimulation, and total dosage of Gn among the four groups (*p* > 0.05).

### 3.2. Comparison of Fertilization after Different Doses of hCG Supplementation in a GnRH-Agonist Trigger Protocol

As shown in Table 2, the GnRH-a + 1000 IU hCG, GnRH-a + 2000 IU hCG, and GnRH-a + 3000 IU hCG groups had more oocytes retrieved, embryos, high-quality embryos, and a higher rate of high-quality embryos than the GnRH-a group (*p* < 0.05). Further analyses demonstrated more oocytes retrieved, embryos, high-quality embryos, and a higher rate of high-quality embryos in the GnRH-a + 1000 IU hCG group than the GnRH-a + 2000 IU hCG and GnRH-a + 3000 IU hCG groups (*p* < 0.05).

### 3.3. The Incidence of OHSS after Different Doses of hCG Supplementation in a GnRH-Agonist Trigger Protocol

No moderate and severe OHSS cases occurred in the GnRH-a and GnRH-a + 1000 IU hCG groups. The incidence rate of moderate and severe OHSS in the GnRH-a + 2000 IU hCG and GnRH-a + 3000 IU hCG groups were 12.96% (7/54) and 11.67% (7/60). The incidence rate of moderate and severe OHSS was remarkably lower in the GnRH-a group and GnRH-a + 1000 IU hCG groups than in the GnRH-a + 2000 IU hCG and GnRH-a + 3000 IU hCG groups; no significant difference was noted between the GnRH-a group and GnRH-a + 1000 IU hCG groups and between the GnRH-a + 2000 IU hCG and GnRH-a + 3000 IU hCG groups (*p* < 0.05, Table 2).

### 3.4. Clinical Outcomes of the First Frozen-Thawed Transfer Cycles

No significant difference was observed in the application of endometrial preparation protocols among the four groups. The clinical pregnancy rates in the GnRH-a, GnRH-a + 1000 IU hCG, GnRH-a + 2000 IU hCG, and GnRH-a + 3000 IU hCG groups were 52.38% (22/42), 57.14% (28/49), 61.11% (33/54), and 60.00% (36/60), respectively. The GnRH-a + 1000 IU hCG, GnRH-a + 2000 IU hCG, and GnRH-a + 3000 IU hCG groups had a higher clinical pregnancy rate than the GnRH-a group, showing no significant difference (*p* > 0.05). The abortion rates in the GnRH-a, GnRH-a + 1000 IU hCG, GnRH-a + 2000 IU hCG, and GnRH-a + 3000 IU hCG groups were 22.73% (5/22), 0.00% (0/28), 3.03% (1/33), and 2.78% (1/35), respectively. The GnRH-a + 1000 IU hCG, GnRH-a + 2000 IU hCG, and GnRH-a + 3000 IU hCG groups had a lower abortion rate than the GnRH-a group (*p* < 0.05, Table 3); no significant difference in the abortion rate was noted among the GnRH-a + 1000 IU hCG group, the GnRH-a + 2000 IU hCG, and GnRH-a + 3000 IU hCG groups (*p* > 0.05).

## 4. Discussion

In the process of ovulation induction, the selection and dose of trigger drugs attach great importance. hCG, as a substitute for LH, induces luteinization of granulosa cells and final maturation of oocytes, which has been commonly and successfully used for decades [19]. However, the application of hCG is associated with the high risk of OHSS due to its high affinity for LH receptor and long half-life [20]. OHSS refers to iatrogenic complications caused by ovarian stimulation, which occurs in the luteal phase or early pregnancy. Although the prevalence of severe OHSS was reported to be between 0.5 and 5%, it has potentially fatal consequences, such as renal failure, hypovolemic shock, thromboembolic events, acute respiratory distress syndrome, and even death [21, 22]. Furthermore, females with high ovarian response, relating to the abnormal sensitivity of the ovary to gonadotropin, are prone to run the risk of OHSS [23]. OHSS remains a serious problem for specialists dealing with infertility.

In recent years, with the development of reproductive medicine technology, clinical ovulation induction programs are more diversified and individualized. It has been observed the GnRH-a can effectively lower the incidence of OHSS but may result in the reduction of egg retrieval rate and egg maturation rate [24]. The trigger drugs, which can reduce the occurrence of OHSS and improve pregnancy outcome, as well as the optimal dose of drugs, have been concerned by reproductive medicine experts. In view of the advantages and disadvantages of hCG and GnRH-a trigger, this study intends to analyze the dual trigger protocol of GnRH-a and hCG in COH scheme, to explore the effect of GnRH-a trigger with different doses of hCG on assisted reproductive pregnancy outcome and the incidence of OHSS in the females with high ovarian response.

Itskovitz-Eldor et al. [25] first described in 2000 that, as for the females with a high risk of OHSS, the adoption of GnRH antagonist protocol with using a single bolus of GnRH-a achieved a 50% pregnancy rate without any symptoms of OHSS. This protocol for ovulation induction has been proven by another study, which pointed out the OHSS can be eliminated by using GnRH and GnRH-a in combination [26]. However, due to the significantly decreased clinical pregnancy rate and increased early abortion rate [27], experts began to focus on improving clinical outcomes through luteal support, including a new method of GnRH-a trigger combined with low-dose hCG. In 2010, Humaidan et al. [28] manifested the protocol of 0.5 mg GnRH-a supplemented with 1500 IU hCG, which proved better pregnancy outcomes, including ongoing pregnancy rate, delivery rate, and early pregnancy loss rate, as well as the zero cases of OHSS. However, in 2013, Seyhan et al. [29] considered that 6 of the 23 females (26%) with high ovarian response developed severe OHSS using the addition of 1500 IU hCG.

In the present study, a total of 205 high ovarian responders were involved and divided into 4 groups. The protocol of 0.2 mg GnRH-a, 0.2 mg GnRH-a + 1000 IU hCG, 0.2 mg GnRH-a + 2000 IU hCG, and 0.2 mg GnRH-a + 3000 IU hCG was applied to the four groups, respectively. The basic information of females in the four groups was not significantly different in terms of mean age, infertility duration, infertility causes, basal FSH, basal LH, basal E2, AFC, duration of Gn stimulation, and total dosage of Gn, which is comparable. Regarding fertilization, we found that the GnRH-a group had fewer oocytes retrieved, embryos, high-quality embryos, and a lower rate of high-quality embryos than the remaining three groups, in which hCG was used in different doses. Furthermore, it was observed the females using GnRH-a supplemented 1000 IU hCG achieved better oocytes retrieved, high-quality embryos, and rate of high-quality embryos than the supplementation of 2000 IU hCG and 3000 IU hCG. Our findings were similar to another research, which observed the poor responders undergoing IVF-ET cycle, Haas et al. [30] indicated that compared to the patients in the hCG trigger and the GnRH-a trigger groups, the patients in the double trigger group (GnRH-a and hCG) had a significantly higher number of top-quality embryos and pregnancy rate. Combined with our above results, it could be suggested that the dual trigger protocol of GnRH-a and hCG is suitable for the poor responders and high ovarian responders undergoing COH. Orvieto [31] also suggested better reproductive outcomes, including oocyte, embryos quality, and luteal phase, occurred in the patients at risk to develop severe OHSS by application of GnRH-a trigger with 1500 IU hCG. Kasum et al. comprehensively analyzed the role of GnRH-a combined with reduced or standard dose hCG in inducing final oocyte maturation in the IVF-ET cycle. The use of GnRH-a and reduced doses of hCG (1000–2500 IU) in high ovarian responders improved luteal support, increased pregnancy rate, and reduced the risk of OHSS [32]. According to the data in this study, we observed no moderate and severe OHSS cases occurred in the patients using GnRH-a trigger alone and dual trigger (GnRH-a and 1000 IU hCG). However, the two groups with GnRH-a + 2000 IU hCG and GnRH-a + 3000 IU hCG, respectively, revealed a high incidence rate of moderate and severe OHSS. To further investigate the clinical outcomes in the patients receiving different trigger protocols, the clinical pregnancy rates and abortion rates were analyzed. It was indicated the GnRH-a group was with a lower rate of clinical pregnancy and higher abortion rate than those using GnRH-a with hCG. The findings were close to another study [33] revealing that, in the patients with high ovarian response, the simultaneous administration of GnRH-a and hCG (1,000 to 2,500 IU) has been confirmed as an effective and safe trigger protocol, which achieved sustained pregnancy and reduced the risk of OHSS. In general, GnRH-a 0.2 mg was adopted due to a large number of follicles in the high response population, who might need relatively more LH to promote follicular maturation. Although different doses of hCG have been reported in many studies abroad, the application dose of hCG (1000 IU, 2000 IU, 3000 IU) we used is associated with the weight of the Asian human body.

Taken together, GnRH-a trigger promotes oocyte maturation by releasing FSH and LH, which reduces the risk of OHS. However, it has an obvious deficiency in luteal support function due to the short half-life of LH, resulting in fewer numbers of oocytes retrieved and fewer high-quality embryos. The application of GnRH-a trigger with hCG supplement achieved better clinical outcomes, involving more high-quality embryos and oocytes retrieved, high clinical pregnancy rate, and low abortion rate. Furthermore, compared to the supplement use of 2000 IU hCG and 3000 IU hCG, the addition of 1000 IU hCG in high ovarian responders minimized the risk of OHSS. However, some limitations, including small sample capacities and lacks of fresh cycle transplantation, were involved in the study, which could lower the accuracy of experimental data. Anyway, this study provides a clinical reference for improving the success rate of IVF-ET treatment and preventing and reducing the occurrence of OHSS.

## Figures and Tables

**Figure 1:** Participant flow and study design.

**Table 1:** The information about basal FSH, basal LH, basal estradiol, AFC, duration of Gn stimulation, and total dosage of Gn in the GnRH-a, GnRH-a + 1000 IU hCG, GnRH-a + 2000 IU hCG, and GnRH-a + 3000 IU hCG groups.

Item	GnRH-a	GnRH-a + 1000 IU hCG	GnRH-a + 2000 IU hCG	GnRH-a + 3000 IU hCG	*p*
Cycles	42	49	54	60	
Basal FSH (U/L)	7.69 ± 2.15	7.89 ± 3.04	7.47 ± 2.55	7.61 ± 2.87	0.885
Basal LH (U/L)	4.66 ± 1.58	4.84 ± 1.72	5.00 ± 1.77	4.55 ± 1.60	0.510
Basal estradiol (pmol/L)	182.22 ± 90.29	180.05 ± 91.33	179.65 ± 89.74	184.39 ± 98.04	0.993
AFC	20.47 ± 1.75	20.88 ± 2.02	21.03 ± 1.69	20.58 ± 1.59	0.356
Duration of Gn stimulation (d)	9.87 ± 1.76	9.69 ± 1.80	9.45 ± 1.78	9.47 ± 1.70	0.607
Total dosage of Gn (U)	1642.55 ± 523.47	1603.45 ± 488.07	1592.47 ± 479.39	1732.08 ± 605.89	0.486

**Table 2:** Comparison of fertilization and incidence of OHSS in the GnRH-a, GnRH-a + 1000 IU hCG, GnRH-a + 2000 IU hCG, and GnRH-a + 3000 IU hCG groups.

Item	GnRH-a	GnRH-a + 1000 IU hCG	GnRH-a + 2000 IU hCG	GnRH-a + 3000 IU hCG
Cycles	42	49	54	60
Oocytes retrieved	15.25 ± 3.78	22.35 ± 5.43^ab^	20.26 ± 4.57^a^	19.67 ± 5.08^a^
Embryos	9.51 ± 3.01	15.63 ± 6.20^ab^	12.57 ± 5.26^a^	11.35 ± 4.79^a^
High-quality embryos	5.26 ± 1.76	10.38 ± 4.51^ab^	8.03 ± 2.31^a^	7.15 ± 2.02^a^
Rate of high-quality embryos (%)	55.31 ± 4.33	66.41 ± 5.79^ab^	63.88 ± 5.11^a^	63.00 ± 5.09^a^
Moderate/severe OHSS (%)	0.00%	0.00%	12.96%	11.67%

^a^ *p* < 0.05 when compared to the GnRH-a group; ^b^*p* < 0.05 when compared to the GnRH-a + 3000 IU hCG group.

**Table 3:** Clinical outcomes of the first frozen-thawed transfer cycles in the GnRH-a, GnRH-a + 1000 IU hCG, GnRH-a + 2000 IU hCG, and GnRH-a + 3000 IU hCG groups.

Item	GnRH-a	GnRH-a + 1000 IU hCG	GnRH-a + 2000 IU hCG	GnRH-a + 3000 IU hCG
Cycles	42	49	54	60

*Endometrial preparation protocols*				
Hormone replacement cycles	31 (73.81%)	37 (75.51%)	42 (77.78%)	46 (76.67%)
Ovulation induction cycles	2 (4.76%)	3 (6.12%)	2 (3.70%)	2 (3.34%)
Downregulation hormone replacement cycles	9 (21.43%)	9 (18.37%)	10 (18.52%)	12 (19.99%)
Clinical pregnancy rate	22 (52.38%)	28 (57.14%)	33 (61.11%)	36 (60.00%)
Abortion rate	22.73% (5/22)	0.00% (0/28)	3.03% (1/33)	2.78% (1/35)

## Data Availability

The data used to support the findings of this study are included within the article.
